# An Online-Offline Certificateless Signature Scheme for Internet of Health Things

**DOI:** 10.1155/2020/6654063

**Published:** 2020-12-31

**Authors:** Muhammad Asghar Khan, Sajjad Ur Rehman, M. Irfan Uddin, Shibli Nisar, Fazal Noor, Ali Alzahrani, Insaf Ullah

**Affiliations:** ^1^Hamdard Institute of Engineering & Technology, Islamabad 44000, Pakistan; ^2^Department of Electrical Engineering, Namal Institute, Mianwali, Pakistan; ^3^Institute of Computing, Kohat University of Science and Technology, Kohat 26000, Pakistan; ^4^Department of Electrical Engineering, National University of Sciences and Technology (NUST), Islamabad 44000, Pakistan; ^5^Department of Computer Science and Information Systems, Islamic University of Madinah, Madinah 400411, Saudi Arabia

## Abstract

The Internet of Health Things (IoHT) is an extended breed of the Internet of Things (IoT), which plays an important role in the remote sharing of data from various physical processes such as patient monitoring, treatment progress, observation, and consultation. The key benefit of the IoHT platform is the ease of time-independent interaction from geographically distant locations by offering preventive or proactive healthcare services at a lower cost. The communication, integration, computation, and interoperability in IoHT are provided by various low-power biomedical sensors equipped with limited computational capabilities. Therefore, conventional cryptographic solutions are not feasible for the majority of IoHT applications. In addition, executing computing-intensive tasks will lead to a slow response time that can deteriorate the performance of IoHT. We strive to resolve such a deficiency, and thus a new scheme has been proposed in this article, called an online-offline signature scheme in certificateless settings. The scheme divides the signing part into two phases, i.e., online and offline. In the absence of a message, the offline phase performs computationally intensive tasks, while lighter computations are executed in the online phase when there is a message. Security analyses and comparisons with the respective existing schemes are carried out to show the feasibility of the proposed scheme. The results obtained authenticate that the proposed scheme offers enhanced security with lower computational and communication costs.

## 1. Introduction

IoHT is an IoT submarket, capable of grouping all medical devices and applications for gathering, analyzing, and exchanging physiological data of patients over the Internet [1]. Patient data can be collected through biomedical sensors and processed via user terminal devices such as computers, smart phones, smart watches, or even a specific embedded device [2]. Patient data may include breathing rate, blood pressure, chest sound, body temperature, respiratory rate, electrocardiogram (ECG), patient position (accelerometer), etc. [3–7]. In addition to medical applications, IoHT can also be used to monitor environmental conditions such as patient-care venues, room status, laboratory shift times, treatment times, and staff-to-patient ratios. The user terminal devices are linked to a gateway via short-range wireless technologies such as Bluetooth Low Energy (BLE), Wi-Fi, and Zigbee. The BLE, however, uses strong features such as moderate data rate, low-power consumption, and unlicensed band, making them the most preferable options for connecting wearable sensor nodes. The gateway may be further connected to a (clinical) server or cloud services via fifth-generation (5G) wireless link for high storage and intensive data processing. In a health information system, patient details can be maintained as electronic health records, which are available to the medical professionals when the patient visits the hospital.

Since a large scale of interactions between biomedical sensors and mobile devices is undertaken on an open wireless channel in IoHT environment, which poses a range of challenges, the most significant of which is the security and privacy of health-related information of patients [8]. To steal or fabricate patient health-related information, an intruder may capture the communication between the sensors and mobile devices. Likewise, with high probability, the attacker may gain access to the disease or health status of the patient. In addition, most devices involved in the IoHT platform have limited computing capabilities and, consequently, fail to perform conventional cryptographic calculations. For example, heavy computations are needed for most of the public key cryptosystems proposed in the literature; therefore, their implementation has not been considered acceptable for IoHT devices. An online-offline approach can be used to address heavy computation issues. When the IoHT devices have reported a message, the online phase is used to perform light computations only, while the offline computations or heavy computations are performed if no message has been recorded by the IoHT devices. Authentication is a major concern for securing IoHT devices. In general, the digital signature is used for authentication in cryptography. Therefore, the digital signature can be used with the online-offline approach for securing IoHT devices. The offline-computed signature value is generated in the offline phase, while the online phase operates with the same offline signature value.

The two basic methods used to validate the public keys are Identity-Based Cryptography (IBC) and Public Key Infrastructure (PKI) in public key cryptosystems. This includes a Certificate Authority (CA) signature, which provides a unique signature link [9]. The CA specifies the public keys with the certificates as defining a participant. However, shortcomings such as distribution, storage, and manufacturing difficulties are associated with PKI systems. Instead, IBC is suggested to decrease the cost of public-key management [10]. The trusted Private Key Generator (PKG) has first-hand data about the participants' private keys with the expense of private key escrow issues [11, 12]. Therefore, certificateless cryptosystem can be used with the signature scheme to accommodate the key escrow problem.

Some computationally hard problems, such as bilinear pairing, Rivest–Shamir–Adleman (RSA), and elliptic curve cryptosystems, usually measure the efficiency of signature schemes. The RSA cryptosystem [13, 14] uses a large key of 1024 bits [15]. Likewise, due to the massive pairing and map-to-point function computation, bilinear pairing is 14.31 times lower than RSA [16]. Similarly, in order to remove the shortcomings of RSA and bilinear pairing, the elliptic curve was introduced [17]. The security hardness and efficiency of elliptic curve cryptography are based on 160-bit keys compared to bilinear pairing and RSA [18]. Despite this, for resource-hungry devices, the 160-bit key is also undesirable and not affordable. Therefore, a new form, the generalization of the elliptic curve, called the hyperelliptic curve was thus suggested [19]. The hyperelliptic curve offers the same degree of protection as the elliptic curve, bilinear pairing, and RSA using 80-bit keys, identity, and certificate size [20, 21]. For energy-constrained IoHT devices, the hyperelliptic curve would be a better option. Therefore, the data generated by the anticipated massive number of biomedical sensors and IoT devices would need to be collected, processed, and analyzed efficiently in real-time to ensure safe and timely management of patient health [22].

Considering the above objectives, a new scheme, called the online-offline certificateless signature scheme, has been introduced for IoHT. The scheme uses the concept of the hyperelliptic curve and is characterized by the small key size. In comparison, it is uncompromisingly identical to the solutions introduced by the elliptical curve method with half key size.

The research study conducted has the following excellent characteristics:

- A lightweight security scheme, namely, online-offline certificateless signature, has been proposed for an IoHT platform.
- The proposed scheme divides the certificateless signature scheme into two phases, i.e., online and offline. Lighter computations are performed when there is a message in the online phase, while the offline phase performs computing-intensive tasks in the absence of a message.
- The scheme uses the hyperelliptic curve cryptography that tackles the limitations faced by IoHT devices such as limited energy and computing capabilities.
- The proposed scheme has shown to be immune to numerous attacks through formal security analysis.
- Our approach offers better efficiency in terms of computational cost and communication overhead when compared to the existing equivalent schemes.

### 1.1. Structure of the Paper

The rest of the article is structured as follows. In Section 2, the relevant work is discussed.  Section 3 includes preliminaries. The proposed online-offline certificateless signature system is introduced in Section 4. Security analysis can be found in Section 5. The cost analysis is provided in Section 6 with current solutions. Concluding remarks are available in Section 7.

## 2. Related Work

In scientific literature, the security and privacy concerns using the online-offline approach have not received ample consideration. Thus, the problems need to be thoroughly investigated. A well-designed security framework would greatly minimize the risk of the data being hacked, regardless of the devilish strategy involved. Some research studies are devoted to addressing IoHT platform data security problems.

The offline-online signature technique was first suggested by Even et al. [23], which is suitable for limited-storage devices. When the message to be signed is known, the execution of their procedure enables the use of the offline mechanism to do moderate computations. After the message is understood to be authenticated, the second phase is carried out electronically. The protection of their method is dependent on the intractability of the large integer factoring mechanism. Their device is protected by chosen messages from attacks. However, their approach is not so successful in practice.

In 2001, to create an effective online-offline signature scheme, Shamir and Tauman [24] used chameleon hash functions based on an ordinary digital signature. In the proposed scheme, the key scale and signature sizes are reduced according to the original scheme. A new type of hash function, called the trapdoor hash function, has been introduced in their model to increase the system security. If the signer repeatedly uses the same hash value to get two signatures on two distinct messages, the recipient can gain a hash collision and use it to retrieve trapdoor information from the signer, which is the secret key of the signer. However, the proposed scheme uses many chameleon hash values for various messages. The main disclosure issue of chameleon hashing is known as this concern.

Yu and Tate [25] suggested an effective online-offline signature scheme that is known to be secure without a random oracle under the RSA assumption. They did not use the hash function at the trapdoor. Therefore, the second key pair did not need to be handled by their scheme and did not have to include in their signature the random commitment attribute. However, the proposed scheme is not affordable for resource-constrained IoHT devices due to the RSA cryptosystem, which is based on hard problems and incurs the high computational cost. Wu et al. [26], using bilinear pairing, suggested a successful online-offline signature scheme. The security of the model is connected to the theoretical Diffie–Hellman assumption in the random oracle model. Addobea et al. [27] also proposed an offline-online signature scheme called the MHCOOS for M-Health devices based on bilinear pairing. However, bilinear pairing involves high pairing and map-to-point function operations, which is not suitable for resource-constrained IoHT devices.

All of the above schemes are based on complex cryptographic techniques, i.e., elliptic curve and bilinear pairing, and thus suffer from high costs of computation and communication overhead. These schemes are thus not compatible with IoHT systems equipped with minimal computing capability. To create a viable IoHT cryptographic solution that needs less computation, there is a critical need to use the state-of-the-art online-offline certificateless signature technique. Our proposed scheme is based on hyperelliptic curve cryptography, which is an advanced version of the elliptic curve. It provides the same degree of protection with the smaller key size as compared to an elliptical curve, bilinear pairing, and modular exponential.

## 3. Preliminaries

### 3.1. Hyperelliptic Curve Discrete Logarithm Problem (**HC** **DL** **P**)

Suppose a given instance of hyperelliptic curve *δ* = *ε*. Then, the HCDLP is to determine *ε* from the given instance.

### 3.2. Threat Model

The security models of the proposed scheme include message *c*, unforgeability against the adversaries called Type 1 adversary (A_1_), and Type 2 adversary (A_2_), respectively. A_1_ is a malicious adversary who has the ability to replace the user's public key besides the system master keys, while A_2_ means an honest-but-curious KGC who knows the system master keys but is not allowed to replace the user's public key. The specific security models under different adversaries are as same as [28] such that unforgeability regarding EUF-CMA-A_1_ and unforgeability regarding EUF-CMA-A_2_.

## 4. Proposed Online-Offline Certificateless Signature Scheme

### 4.1. Network Model

An initiative to incorporate the proposed scheme must be preceded by careful consideration of the following assumptions:

1. Patient data input can be obtained by sensors and analyzed by user terminal devices, such as laptops, tablets, smart watches, or even a particular embedded system
2. Each of the medical sensors and the user terminal are connected through BLE
3. The user terminal can be further linked with the cloud server using 5G, equipped with cloud computing services
4. The medical server presumes the role of administrators
5. The medical server is linked with the local computer in which electronic health records (HER) can be viewed by the medical personnel
6. The HER is stored securely in the database server for future consultations

IoHT can be implemented in various settings, depending on the requirements as shown in Figure 1. The required gadgets are usually included in the medical sensors according to the patient's illness. Using short-range radio transceivers (i.e., BLE), the sensors can be connected with the gateway router. On a frequency band of 2.4 GHz, the BLE works. There are valid reasons for selecting this level of technology. They function, for example, in the unlicensed spectrum and provide fair data rates and consume very low power [29]. The aggregated data from the patient monitoring sensors may be too big to be handled by the local server. It demands a high ability for storage and computing. Fortunately, with its architecture, the emerging fifth-generation (5G) mobile networking introduces multiaccess edge computing (MEC) facility. MEC performs high storage and intensive processing facilities when integrated into an IoHT setting.

### 4.2. Construction of the Proposed Scheme

This section covers the construction of the proposed scheme. Notations used in the proposed scheme are illustrated in Table 1. The proposed scheme can be made from the following computational constructions [28]:

  Setup: the following computations can be used for this phase:
(i) The security parameter *η* can choose by KGC
(ii) It selects a hyperelliptic curve (𝒽𝒸) with field *f*(*n*), where the size of *n* ≥ 2^80^
(iii) Select a 𝒟 devisor from hyperelliptic curve (𝒽𝒸)
(iv) Then, choose three irreversible and collision resistance hash functions *h*_*x*_,  *h*_*y*_,  and *h*_*z*_
(v) KGC picks 𝒬  ∈  {1,2,…,  *n* − 1} as a master key and then computes the public key as *𝒦*=𝒬 · *𝒟*
(vi) KGC produces *ψ* = {𝒦, ℎ𝑥, ℎ𝑦, ℎ𝑧, 𝒟, 𝒽𝒸, (𝑛), 𝑛≥2^80^ as global parameter set and publishes it publicly
  Secret value setting: the participating entity with identity *id*_*i*_ picks *l*_*i*_  ∈  {1,2,…,  *n* − 1}as a secret value and computes *𝒱*_*i*_ = *l*_*i*_ · *𝒟* as a public key
  Partial private key setting: for a participating entity with identity *id*_*i*_*, the* KGC picks *ϑ*_*i*_  ∈  {1,2,…,  *n* − 1}, computes *μ*_*i*_ = *ϑ*_*i*_ · *𝒟*, calculates 𝓌_𝑖_, = *ϑ*_*i*_+𝒬*h*_*x*_(*id*_*i*_, *𝒱*_*i*_, *μ*_*i*_), and sends Γ_*i*_= (𝓌_𝑖_,𝜇_𝑖_) to entity with *id*_*i*_ via secure network
  Private key setting: the participating entity, with identity *id*_*i*_, sets *𝒩*_*i*_=(Γ_*i*_, *l*_*i*_)of its private key.
  Public key setting: the participating entity, with identity *id*_*i*_, set_s_ *𝒵*_*i*_=(*𝒱*_*i*_, *μ*_*i*_) of its public key.
  Certificateless online/offline signature: the sender computations can be divided into the following two substeps, e.g., Online and Offline.
  Offline phase: this part will be run over the server that is equipped with high resources and the construction step is carried out as follows:
(i) It picks ∈ {1,2,…,  *n* − 1} and computes 𝓉= = 𝒹·*𝒱*_*s*_
  (ii)Compute 𝒫=ℎ𝑦 (𝑖𝑑𝑠, 𝜇𝑠, 𝑚, 𝓉) and 𝒳=ℎ𝑧 (𝑖𝑑𝑠, 𝒱𝑠, 𝑚, 𝓉)
(iii) Then, it gives (𝒹, 𝓉, 𝒫, 𝒳) to the sensor nodes
  Online phase: this part will be run on the sensor nodes and the construction step consists as follows:
  (i)Compute *𝒮*= *l*_*s*_·𝒹−(*l*_*s*_ · *𝒳* + *𝒫* ·  𝓌𝑠)
(ii) Set *ϕ*=(*t*, *S*) as a signature and send it to the receiver
  Certificateless online/offline signature verification: upon reception *ϕ*, a receiver can verify *𝒮* as follows:
(i) Compute *P*=*h*_*y*_(*id*_*s*_, *μ*_*s*_, *m*, *t*) and *χ*=*h*_*z*_(*id*_*s*_, *𝒱*_*s*_, *m*, *t*)
(ii) Then, it checks if  *S* · *D*=*t* · *χ𝒱*_*s*_ − *𝒫*(*μ*_*s*_+*h*_*x*_(*id*_*s*_, *𝒱*_*s*_, *μ*_*s*_)*𝒦*) holds

### 4.3. Correctness

The verifier/receptionist can verify the signature if the following computation is successfully processed:

So, if *P*=*h*_*y*_(*id*_*s*_, *μ*_*s*_, *m*, *t*) and *X*=*h*_*z*_(*id*_*s*_, *𝒱*_*s*_, *m*, *t*), we acquire

(1) $$\begin{array}{c} S.D=\left(\;l_{s}\cdot d-\left(\;l_{s}\;\cdot X\;+\;P\cdot w_{s}\right)\right)D\\ =\left(\;l_{s}\cdot d\cdot D-\left(\;l_{s}\cdot X\;+\;P\cdot w_{s}\right)\right)D\\ =\left(V_{s}\right.\cdot d-\left(\;l_{s}\cdot X\;+\;P\cdot w_{s}\right)D\\ =\left(t-\left(\;l_{s}\cdot \;X\right)\right.D-\left(P.w_{s}\right)D\\ =\left(t-\left(\;l_{s}\cdot X\cdot D\;\right)\right.-\left(P\cdot w_{s}\right)D\\ =\left(t-\left(V_{s}\cdot X\;\right)-\left(P\cdot \left(\vartheta_{s}+\;Qh_{x}\left(id_{s},V_{s},\mu_{s}\right)\right)\right.D\right)\\ =\left(t-\left(V_{s}\cdot X\;\right)-\left(P\cdot \;\left(\vartheta_{s}.D+\;Q\cdot Dh_{x}\left(id_{s},V_{s},\mu_{s}\right)\right)\;\right.\right)\\ =\left(t-\left(V_{s}\cdot X\;\right)\right.-\left(P\cdot \left(\vartheta_{s}\cdot D+\;Q\cdot Dh_{x}\left(id_{s},V_{s},\mu_{s}\right)\right)\right.\;\\ =\left(t-\left(V_{s}.X\;\right)\right.-\left(P\cdot \left(\mu_{s}+h_{x}\left(id_{s},V_{s},\mu_{s}\right)K\right)\right.\cdot \end{array}$$

This validates the correctness of the proposed scheme.

## 5. Security Analysis

The purpose of this section is to explain the usefulness of the suggested method in resisting attacks.

**Theorem 1 .**

The proposed scheme resists against an adaptive chosen message attack, if an adversary A_1_would not be able to solve the hyperelliptic curve discrete logarithm problem (HECDLP).

**Proof**

Suppose there is a challenger *ζ* which helps *A*_1_ to extract  *ℓ* from the given instance *f*=*ℓ* · *𝒟* of HECDLP. Further, to figure out HECDLP, *ζ* can set the master key secret key as 𝒬=*ℓ* and master public key as *𝒦*=*ℓ* · *𝒟*. Then, *ζ* generates *ψ* as a global parameter set and four empty lists (*L*_ *h*_*x*__, *L*_ *h*_*y*__, *L*_ *h*_*z*__, *L*_*k*_) for holding the value of *h*_*x*_, *h*_*y*_, *h*_*z*_, and keys.

  Create (**id**_**i**_): after reception, Create *id*_*i*_ query, *ζ* selects  *α*_*i*_, *β*_*i*_, *l*_*i*_ ∈  {1,2, .. … .,  *n* − 1} and sets *h*_*x*_(*id*_*i*_, *𝒱*_*i*_, *μ*_*i*_)=−*β*_*i*_,  *𝒱*_*i*_=*l*_*i*_.*𝒟*, and *μ*_*i*_=*β*_*i*_.*𝒦* −  *α*_*i*_.*𝒟*. Then, *ζ* answers in the following two steps:
(i) If *id*_*i*_ ≭ *id*_*s*_, with the identity **id**_**i**_, *ζ* outputs will be (Γ_*i*_=*v*_*i*_, *μ*_*i*_), *𝒩*_*i*_=(⊥, *l*_*i*_), and  *𝒵*_*i*_=(*𝒱*_*i*_, *μ*_*i*_), respectively.
(ii) If *id*_*i*_ ≭ *id*_*s*_, with the identity **id**_**i**_, *ζ* outputs will be (Γ_*i*_=*v*_*i*_, *μ*_*i*_), *𝒩*_*i*_=(Γ_*i*_, *l*_*i*_), and  *𝒵*_*i*_=(*𝒱*_*i*_, *μ*_*i*_), respectively.
  Thus, *ζ* included (*id*_*i*_, *𝒱*_*i*_, *μ*_*i*_, *β*_*i*_) into *L*_ *h*_*x*__ and (*id*_*i*_, Γ_*i*_, *𝒩*_*i*_,  *𝒵*_*i*_) into *L*_*k*_.
  Hash queries ( *h*_*x*_, *h*_*y*_, *h*_*z*_): after reception, Hash queries ( *h*_*x*_, *h*_*y*_, *h*_*z*_), *ζ* searches for the values  Ω_*i*_, *𝒫*_*i*_, *𝒳*_*i*_ in lists *L*_ *h*_*x*__, *L*_ *h*_*y*__, *L*_ *h*_*z*__; if it finds in these lists then retunes to *A*_1_; otherwise, the values  Ω_*i*_, *𝒫*_*i*_, *𝒳*_*i*_ for each Hash query will select by *ζ* in a random manner and send it to the *A*_1_.
  Secret value setting queries: after reception, this query, then, (*ζ*) answers in the following two steps:
(i) If *id*_*i*_=*id*_*s*_, *ζ* aborts the process.
(ii) If *id*_*i*_ ≭ *id*_*s*_, *ζ* will look for (*id*_*i*_, Γ_*i*_, *𝒩*_*i*_,  *𝒵*_*i*_) in *L*_*k*_; if such a tuple is found, then it results in *l*_*i*_; otherwise, *ζ* calls Create *id*_*i*_ query and gets (*id*_*i*_, Γ_*i*_, *𝒩*_*i*_,  *𝒵*_*i*_) and then sends *l*_*i*_ to *A*_1_.
  Partial private key setting queries: after reception, this query, then, (*ζ*) answers in the following two steps:
(i) If *id*_*i*_=*id*_*s*_, *ζ* aborts the process.
(ii) If *id*_*i*_ ≭ *id*_*s*_, *ζ* will look for (*id*_*i*_, Γ_*i*_, *𝒩*_*i*_,  *𝒵*_*i*_) in *L*_*k*_; if such a tuple is found, then it sends Γ_*i*_to *A*_1_.
  Public key setting queries: after reception, this query, then, (*ζ*) answers in the following two steps:
(i) If *id*_*i*_=*id*_*s*_, *ζ* aborts the process.
(ii) If *id*_*i*_ ≭ *id*_*s*_, *ζ* will look for (*id*_*i*_, Γ_*i*_, *𝒩*_*i*_,  *𝒵*_*i*_) in *L*_*k*_; if such a tuple is found, then it results in *𝒵*_*i*_=(*𝒱*_*i*_, *μ*_*i*_); otherwise, *ζ* calls Create *id*_*i*_ query and gets (*id*_*i*_, Γ_*i*_, *𝒩*_*i*_,  *𝒵*_*i*_) and then sends  *𝒵*_*i*_=(*𝒱*_*i*_, *μ*_*i*_) to *A*_1_.
  Public key replacement queries: after reception, this query, then, (*ζ*) will look for (*id*_*i*_, Γ_*i*_, *𝒩*_*i*_,  *𝒵*_*i*_) in *L*_*k*_ and replace  *𝒵*_*i*_ by  *𝒵*_*i*_^*∗*^ and include (*id*_*i*_, Γ_*i*_, *𝒩*_*i*_,  *𝒵*_*i*_^*∗*^) into *L*_*k*_. So, *ζ* sets *w*_*i*_=⊥ and *𝒩*_*i*_=*|*⊥.
  Certificateless online/offline signature queries: after reception, this query, then, (*ζ*) checks. If *id*_*i*_=*id*_*s*_, then it aborts the process; otherwise, it will perform the following steps:
(i) *ζ* first gets access to *L*_ *h*_*y*__, *L*_ *h*_*z*__, and *L*_*k*_.
  Offline phase:
(ii) It picks  *d*_*i*_ ∈  {1,2,…,  *n* − 1} and computes *d*_*i*_=*d*_*i*_ · *V*_*s*_.
  Online phase:
(iii) Compute *𝒮*_*i*_= *l*_*i*_.*d* _*i*_ − ( *l*_*i*_. *𝒳*_*i*_ + *𝒫*_*i*_. *w*_*i*_) and it results as a signature Φ=*t*_*i*_, *S*_*i*_.
  Certificateless online/offline signature verification query: after reception, this query, then, (*ζ*) checks. If *id*_*i*_=*id*_*s*_, then it aborts the process; otherwise, it will perform the certificateless online/offline signature verification algorithm for the verifications of signature.
  Forgery: at the end, *A*_1_ results a lawful signature (Φ=*t*_*i*_, *S*_*i*_). If *id*_*i*_=*id*_*s*_, *ζ* aborts the process; otherwise, *ζ* checks for a list *L*_ *h*_*x*__, and according to forking lemma , it generates another signature Φ^*∗*^=(*𝒮*_*i*_^*∗*^,  *t*_*i*_). So, we have *𝒮* · *𝒟*= *t*_*s*_ − *X* ·  *𝒱*_*s*_ − *𝒫*_*s*_. (*μ*_*s*_+ Ω_*s*_*𝒦*) and *𝒮*_*s*_^*∗*^ · *𝒟*= *t*_*s*_ − *X* ·  *𝒱*_*s*_ − *𝒫*_*s*_^*∗*^. (*μ*_*s*_+ Ω_*s*_*𝒦*). We suppose that *μ*_*s*_=*β*_*s*_ · *𝒦*+ *α*_*s*_ · *𝒟* and *𝒦* =  *ℓ* · *𝒟*. So, when the subtractions between these two equations are performed, then we can get the following computations:

(2) $$\begin{array}{c} S_{i}^{*}-S\cdot D=\left(t_{s}-X\cdot \;V_{s}-P_{s}^{*}\cdot \;\left(\mu_{s}+\;\Omega_{s}K\right)\right)\left(t_{s}-X\cdot \;-\;V_{s}-P_{s}\cdot \;\left(\mu_{s}+\;\Omega_{s}K\right)\right),\\ S_{i}^{*}\cdot D-S\cdot D=t_{s}-X\;V_{s}-P_{s}^{*}\cdot \;\left(\mu_{s}+\;\Omega_{s}K\right)-\;t_{s}-X\cdot \;V_{s}+P_{s}\cdot \;\left(\mu_{s}+\;\Omega_{s}K\right),\\ S_{i}^{*}\cdot D-S\cdot D=P_{s}\cdot \;\left(\mu_{s}+\;\Omega_{s}K\right)-P_{s}^{*}\cdot \;\left(\mu_{s}+\;\Omega_{s}K\right),\\ \left(S_{i}^{*}-S\right)\cdot D-\left(P_{s}-P_{s}^{*}\right)\;\alpha_{s}\cdot D=\left(P_{s}\right.-P_{s}^{*}\;\left(\beta_{s}+\;\Omega_{s}\right)\ell \cdot D,\\ \left(\left(S_{i}^{*}-S\right)-\left(P_{s}-P_{s}^{*}\right)\;\alpha_{s}\right)\cdot D=\left(P_{s}-P_{s}^{*}\right)\;\left(\beta_{s}+\;\Omega_{s}\right)\ell \cdot D,\\ \left(\left(S_{i}^{*}-S\right)-\left(P_{s}-P_{s}^{*}\right)\;\alpha_{s}\right)=\left(P_{s}-P_{s}^{*}\right)\;\left(\beta_{s}+\;\Omega_{s}\right)\ell \;,\\ \left(\left(S_{i}^{*}\left.-S\right)-\left(P_{s}-P_{s}^{*}\right)\;\alpha_{s}\right)/\left(P_{s}-\left.P_{s}^{*}\right)\;\left(\beta_{s}+\;\Omega_{s}\right.\right)\right)=\ell . \end{array}$$

So, *A*_1_ can solve HECDLP as *ℓ*=((*𝒮*_*i*_^*∗*^ − *𝒮*) − (*𝒫*_*s*_ − *𝒫*_*s*_^*∗*^) *α*_*s*_)/(*𝒫*_*s*_ − *𝒫*_*s*_^*∗*^) (*β*_*s*_+ Ω_*s*_), with the help of challenger *ζ*.

### 5.1. Probability Analysis

Here, we define the following probability events:

- The winning probability of Create query must be greater than (1 − *Q*_*h*_*x*__ *Q*_create_/*n* )
- The succeeded probability of  *h*_*y*_ must be greater than (1 −  *Q*_*h*_*y*__/*n*)
- The succeeded probability of  *h*_*z*_ must be greater than (1 −  *Q*_*h*_*y*__/*n*)
- The succeeded probability of certificateless online/offline signature queries must be greater than ( *Q*_*s*_/*n*)
- *id*_*i*_=*id*_*s*_ satisfies with probability (1/*Q*_create_)

Note that  *Q*_create_,  *Q*_*h*_*x*__,  *Q*_*h*_*y*__, *Q*_*h*_*z*__, and  *Q*_*s*_ represent Create queries and Hash queries to *h*_*x*_,  *h*_*y*_,  *h*_*z*_, and certificateless online/offline signature queries, respectively.

So, overall advantage of *A*_1_ is towards its success as *ξ*^*∗*^ ≥ (1 −  *Q*_*h*_*x*__ *Q*_create_/*n*)(1 −  *Q*_*h*_*y*__/*n*)(1 −  *Q*_*h*_*z*__/*n*)( (1/ *Q*_create_)( *Q*_*s*_/*n*).

**Theorem 2 .**

By using the random oracle model, the proposed scheme resists against an adaptive chosen message attack, if an adversary A_2_would not be able to solve the hyperelliptic curve discrete logarithm problem (HECDLP).

**Proof**

Suppose there is a challenger *ζ* which helps *A*_1_ to extract  *ℓ* from the given instance *f*=*ℓ* · *𝒟*of HECDLP. Further, to figure out HECDLP, *ζ* picks *b* and sets master public key as *𝒦*=*b* · *𝒟*. Then, *ζ* generates *ψ* as a global parameter set, and similar to Theorem 1, it picks four empty lists (*L*_ *h*_*x*__, *L*_ *h*_*y*__, *L*_ *h*_*z*__, *L*_*k*_) for holding the value of *h*_*x*_, *h*_*y*_, *h*_*z*_, and keys.

  Create (*id*_*i*_): after reception, Create *id*_*i*_ query, *ζ* answers in the following steps:
(i) If *id*_*i*_=*id*_*s*_, *ζ* selects  *α*_*i*_, Ω_*i*_ ∈  {1,2,…,  *n* − 1} and sets *h*_*x*_(*id*_*i*_, *𝒱*_*i*_, *μ*_*i*_)=Ω_*i*_,  *𝒱*_*i*_=*ℓ* · *𝒟*, *w*_*i*_=*α*_*i*_+*b*Ω_*i*_, and *μ*_*i*_= *α*_*i*_ · *𝒟*. So, it produces (Γ_*i*_=*w*_*i*_, *u*_*i*_),  *𝒩*_*i*_=(Γ_*i*_, ⊥), and  *𝒵*_*i*_=(*𝒱*_*i*_, *μ*_*i*_), respectively.
(ii) If 𝒊𝒅_𝒊_ ≭ 𝒊𝒅_𝒊_, *ζ* selects  *α*_*i*_, *l*_*i*_, Ω_*i*_ ∈  {1,2,…,  *n* − 1} and sets *h*_*x*_(*id*_*i*_, *𝒱*_*i*_, *μ*_*i*_)=Ω_*i*_,  *𝒱*_*i*_=*l*_*i*_.*𝒟*, *w*_*i*_=*α*_*i*_*b*Ω_*i*_, and *μ*_*i*_= *α*_*i*_.*𝒟*.
  Thus, *ζ* included (*id*_*i*_, *𝒱*_*i*_, *μ*_*i*_, Ω_*i*_) into *L*_ *h*_*x*__ and (*id*_*i*_, Γ_*i*_, *𝒩*_*i*_,  *𝒵*_*i*_) into *L*_*k*_.
  Hash queries ( **h**_**x**_, **h**_**y**_, **h**_**z**_): these are the same as performed in Theorem 1.
  Secret value setting queries: after reception, this query, then, (*ζ*) answers in the following two steps.
(i) If **id**_**i**_=**id**_**s**_, *ζ* aborts the process.
(ii) If 𝒊𝒅_𝒊_ ≭ 𝒊𝒅_𝒊_, *ζ* will look for (*id*_*i*_, Γ_*i*_, *𝒩*_*i*_,  *𝒵*_*i*_) in *L*_*k*_; if such a tuple is found, then it results in *l*_*i*_; otherwise, *ζ* calls Create *id*_*i*_ query and gets (*id*_*i*_, Γ_*i*_, *𝒩*_*i*_,  *𝒵*_*i*_) and then sends *l*_*i*_ to *A*_2_.
  Partial private key setting queries: after reception, this query, then, (*ζ*) answers in the following two steps:
(i) If **id**_**i**_=**id**_**s**_, *ζ* aborts the process.
(ii) If 𝒊𝒅_𝒊_ ≭ 𝒊𝒅_𝒊_, *ζ* will look for (*id*_*i*_, Γ_*i*_, *𝒩*_*i*_,  *𝒵*_*i*_) in *L*_*k*_; if such a tuple is found, then it sends Γ_*i*_to *A*_2_.
  Public key setting queries: after reception, this query, then, (*ζ*) answers in the following two steps:
(ii) If **id**_**i**_=**id**_**s**_, *ζ* aborts the process.
(iii) If 𝒊𝒅_𝒊_ ≭ 𝒊𝒅_𝒊_, *ζ* will look for (*id*_*i*_, Γ_*i*_, *𝒩*_*i*_,  *𝒵*_*i*_) in *L*_*k*_; if such a tuple is found, then it results in  *𝒵*_*i*_=(*𝒱*_*i*_, *μ*_*i*_); otherwise, *ζ* calls Create *id*_*i*_ query and gets (*id*_*i*_, Γ_*i*_, *𝒩*_*i*_,  *𝒵*_*i*_) and then sends  *𝒵*_*i*_=(*𝒱*_*i*_, *μ*_*i*_) to *A*_2_.
  Certificateless online/offline signature queries: after reception, this query, then, (*ζ*) checks. If **id**_**i**_=**id**_**s**_, then it aborts the process; otherwise, it will perform the following steps:
(i) *ζ* first gets access to *L*_ *h*_*y*__, *L*_ *h*_*z*__, and *L*_*k*_.
  Offline phase:
(i) It picks  *d*_*i*_ ∈  {1,2,…,  *n* − 1} and computes *t*_*i*_=*d*_*i*_ · *𝒱*_*s*_.
  Online phase:
(ii) Compute *𝒮*_*i*_= *l*_*i*_ · *d*_*i*_ − ( *l*_*i*_ ·  *X*_*i*_ + *𝒫*_*i*_.·*w*_*i*_) and it results as a signature 𝛷 = (𝓉_𝑖_, 𝒮_𝑖_).
  Certificateless online/offline signature verification query: after reception, this query, then, (*ζ*) checks. If *id*_*i*_=*id*_*s*_, then it aborts the process; otherwise, it will perform the certificateless online/offline signature verification algorithm for the verifications of signature.
  Forgery: at the end, *A*_1_ results in a lawful signature *ϕ*= (𝓉_𝑖_,  *𝒮*_*i*_). If *id*_*i*_=*id*_*s*_, *ζ* aborts the process; otherwise, *ζ* checks for a list *L*_ *h*_*x*__, and according to forking lemma , it generates another signature Φ^*∗*^=(*𝒮*_*i*_^*∗*^,  *t*_*i*_). So, we have *𝒮* · *𝒟*= *t*_*s*_ − *X* ·  *𝒱*_*s*_ − *𝒫*_*s*_. (*μ*_*s*_+ Ω_*s*_*𝒦*) and *𝒮*_*i*_^*∗*^ · *𝒟*= *t*_*s*_ − *X* ·  *𝒱*_*s*_ − *𝒫*_*s*_^*∗*^. (*μ*_*s*_+ Ω_*s*_*𝒦*). We suppose that *μ*_*s*_=*β*_*s*_ · *𝒦*+ *α*_*s*_ · *𝒟* and *𝒦* =  *ℓ* · *𝒟*. So, when the subtractions between these two equations are performed, then we can get the following computations:

(3) $$\begin{array}{c} S_{i}^{*}-S\cdot D=\left(t_{s}-X\cdot \;V_{s}-P_{s}^{*}\cdot \;\left(\mu_{s}+\;\Omega_{s}K\right)\right)\left(t_{s}-X\cdot \;-\;V_{s}-P_{s}\cdot \;\left(\mu_{s}+\;\Omega_{s}K\right)\right),\\ S_{i}^{*}\cdot D-S\cdot D=t_{s}-XV_{s}-P_{s}^{*}\cdot \;\left(\mu_{s}+\;\Omega_{s}K\right)-\;t_{s}-X\cdot \;V_{s}+P_{s}\cdot \;\left(\mu_{s}+\;\Omega_{s}K\right),\\ S_{i}^{*}\cdot D-S\cdot D=P_{s}\cdot \;\left(\mu_{s}+\;\Omega_{s}K\right)-P_{s}^{*}\cdot \;\left(\mu_{s}+\;\Omega_{s}K\right),\\ \left(S_{i}^{*}-S\right)\cdot D-\left(P_{s}-P_{s}^{*}\right)\;\alpha_{s}\cdot D=\left(P_{s}\right.-P_{s}^{*}\;\left(\beta_{s}+\;\Omega_{s}\right)\ell \cdot D,\\ \left(\left(S_{i}^{*}-S\right)-\left(P_{s}-P_{s}^{*}\right)\;\alpha_{s}\right)\cdot D=\left(P_{s}-P_{s}^{*}\right)\;\left(\beta_{s}+\;\Omega_{s}\right)\ell \cdot D,\\ \left(\left(S_{i}^{*}-S\right)-\left(P_{s}-P_{s}^{*}\right)\;\alpha_{s}\right)=\left(P_{s}-P_{s}^{*}\right)\;\left(\beta_{s}+\;\Omega_{s}\right)\ell \;,\\ \left(\left(S_{i}^{*}\left.-S\right)-\left(P_{s}-P_{s}^{*}\right)\;\alpha_{s}\right)/\left(P_{s}-\left.P_{s}^{*}\right)\;\left(\beta_{s}+\;\Omega_{s}\right.\right)\right)=\ell . \end{array}$$

So, *ℓ*=(*𝒮*_*i*_^*∗*^ − *𝒮*)/(*𝒳*^*∗*^ − *𝒳*) as the solution of HECDLP.

The probability analysis is same as Theorem 1 and as follows:

The utilized advantages of *A*_2_ towards its success are as follows:

*ξ* ^*∗*^ ≥ (1 −  *Q*_*h*_*x*__ *Q*_create_/*n*)(1 −  *Q*_*h*_*y*__/*n*)(1 −  *Q*_*h*_*z*__/*n*)( (1/ *Q*_*create*_)( *Q*_*s*_/*n*).

## 6. Cost Analysis

This section contrasts the efficiency of the proposed scheme with the existing equivalents suggested by the schemes of Yu and Tate [25], scheme 1, Yu and Tate [25], scheme 2, Wu et al. [26], and Addobea et al. [27].

### 6.1. Computational Cost

Table 2 displays the key results derived from the analysis. Elliptic curve scalar multiplication and bilinear pairings are used in the existing schemes, all of which are more expensive alternatives. Therefore, we add the multiplication of the hyperelliptic divider. Observations have shown that the time it takes for a single scalar multiplication to be processed differs considerably: elliptic curve point multiplication (ECPM), 0.97 milliseconds; bilinear pairing (P), 14.90 ms; pairing-based point multiplications (BPM), 4.31 ms; and modular exponentiation (E), 1.25 ms [16]. The Multiprecision Integer and Rational Arithmetic C Library (MIRACL) [30] is used to calculate the performance of the proposed system. It checks roughly 1000 times the runtime of specific cryptographic operations. A workstation with the following requirements is used for evaluating simulation results: Intel Core i7-4510U Processor @ 2.0 GHz, 8 GB RAM, and Windows 7 Home Standard 64-bit Operating System [29]. The hyperelliptic curve divisor multiplication (HM) is believed to be 0.48 milliseconds in length due to a smaller key size of 80 bits [31–34]. It is apparent from the results in Tables 2 and 3 that our solution is much more effective in terms of the computational cost as shown in Figure 2.

### 6.2. Communication Cost

This subsection is aimed at discussing the comparison results from the perspective of communication costs. The proposed approach is compared with the existing schemes presented by Yu and Tate [25] scheme 1, Yu and Tate [25] scheme 2, Wu et al. [26], and Addobea et al. [27]. In comparative analysis, the variables, i.e. |**G**| = 1024 bits, |m| = 1024 bits, and |n| = 80 bits, along with the respective values, are depicted in Table 4 and illustrated in Figure 3.

## 7. Conclusion

The Internet of Health Things (IoHT) plays an important role as an extension of the Internet of Things (IoT) in the remote data-sharing of multiple physical processes, such as patient monitoring, treatment progression, observation, and consultation. In IoHT, multiple sensors, actuators, and controllers allow communication, computation, and interoperability, thus providing seamless connectivity with efficient resource utilization. However, for the majority of IoHT implementations, conventional cryptographic methods are not feasible due to the energy constraints of low-power embedded devices. Therefore, we suggested a lightweight security scheme in this article, using the idea of the hyperelliptic curve (HEC), called an online-offline certificateless signature scheme. In the limited key size, the HEC solution is powerful and is also acceptable for IoHT environments. The formal security analysis shows the intensity of the proposed approach in avoiding multiple attacks. In addition, after a comparative comparison with the main existing schemes, the proposed scheme proved to be efficient in terms of both computational and communication costs.

An extension of the proposed scheme is required that offers encryption and digital signature in one go. We also plan to improve the security by adding some other aspects of formal analysis, such as the real-or-random (ROR) for the solutions against different attacks. All these aspects are in the development phase and will be taken into account in our future work.

## Figures and Tables

**Figure 1:** Sample network model of IoHT system.

**Figure 2:** Computational cost (in ms).

**Figure 3:** Communication cost (in bits).

**Table 1:** Notations used.

Notation	Description
*η*	It represents a security parameter
𝒽𝒸	It represents a hyperelliptic curve
*f*(*n*)	It represents a finite field of *n*
*n*	It represents a large prime number belonging to hyperelliptic curve where the size of *n* ≥ 2^80^
𝒟	Divisor on the hyperelliptic curve (𝒽𝒸)
𝒬	Master private key of the system
*𝒦*	Master public key of the system
*ψ*	It represents a global parameter set that can be available publicly in a network
*id*_*s*_, *id*_*r*_	Identity of sender and receiver
Γ_*s*_, Γ_*r*_	They represent partial private key pair for sender and receiver
*𝒩*_*s*_, *𝒩*_*r*_	They represent private key pair for sender and receiver
*𝒵*_*s*_, *𝒵*_*r*_	They represent public key pair for sender and receiver
*𝒮*	Its represents signature
*ϕ*	It represents signature pair
*h*_*x*_, *h*_*y*_, *h*_*z*_	Three irreversible and collision resistance hash functions
⊥	It represents null

**Table 2:** Computational cost.

Schemes	Signing	Verifying	Total
Yu and Tate [25] scheme 1	1*E* + 3BPM	3*E* + 4BPM	4*E* + 7BPM
Yu and Tate [25] scheme 2	2*E* + 3BPM	3*E* + 3BPM	5*E* + 6BPM
Wu et al. [26]	3BPM	2P + 2BPM	2P + 5BPM
Addobea et al. [27]	3 BPM	3P + 4BPM	3P + 7BPM
Proposed	4HM	3HM	7HM

**Table 3:** Computational cost in milliseconds.

Schemes	Signing	Verifying	Total (ms)
Yu and Tate [25] scheme 1	14.18	20.99	35.17
Yu and Tate [25] scheme 2	15.43	16.68	32.11
Wu et al. [26]	12.99	38.42	51.41
Addobea et al. [27]	12.99	61.94	74.93
Proposed	1.92	1.44	3.36

**Table 4:** Communication cost in bits.

Schemes	Communication cost	Communication cost in bits
Yu and Tate [25] scheme 1	3|G| + |m|	4096
Yu and Tate [25] scheme 2	3|G| +|m|	4096
Wu et al. [26]	3|G| + |m|	4096
Addobea et al. [27]	3|G| + |m|	4096
Proposed	2|n| + |m|	1184

## Data Availability

All data generated or analyzed during this study are included in this published article.

## References

[1] Rodrigues J. J. P. C., De Rezende Segundo D. B., Junqueira H. A. (2018). Enabling technologies for the internet of health things. *IEEE Access*.

[2] Riazul Islam S. M., Daehan Kwak D., Humaun Kabir M., Hossain M., Kyung-Sup Kwak K.-S. (2015). The internet of Things for health care: a comprehensive survey. *IEEE Access*.

[3] Catarinucci L., De Donno D., Mainetti L. (2015). An IoT-aware architecture for smart healthcare systems. *IEEE Internet of Things Journal*.

[4] Yin Y., Zeng Y., Chen X., Fan Y. (2016). The internet of things in healthcare: an overview. *Journal of Industrial Information Integration*.

[5] Woo M. W., Lee J. W., Park K. H. (2018). A reliable IoT system for personal healthcare devices. *Future Generation Computer Systems*.

[6] Farahani B., Firouzi F., Chang V., Badaroglu M., Constant N., Mankodiya K. (2018). Towards fog-driven IoT eHealth: promises and challenges of IoT in medicine and healthcare. *Future Generation Computer Systems*.

[7] Firouzi F., Rahmani A. M., Mankodiya K. (2018). Internet-of-things and big data for smarter healthcare: from device to architecture, applications and analytics. *Future Generation Computer Systems*.

[8] Lin X., Lu R., Shen X., Nemoto Y., Kato N. (2009). Sage: a strong privacy preserving scheme against global eavesdropping for ehealth systems. *IEEE Journal on Selected Areas in Communications*.

[9] Ullah S., Marcenaro L., Rinner B. (2019). Secure smart cameras by aggregate-signcryption with decryption fairness for multi-receiver IoT applications. *Sensors*.

[10] Shamir A. (1984). Identity-based cryptosystems and signature schemes. *Proceedings of the of the CRYPTO 1984*.

[11] Kumar P., Kumari S., Sharma V., Sangaiah A. K., Wei J., Li X. (2018). A certificateless aggregate signature scheme for healthcare wireless sensor network. *Sustainable Computing: Informatics and Systems*.

[12] Kumar P., Kumari S., Sharma V., Li X., Sangaiah A. K., Islam S. H. (2019). Secure cls and cl-as schemes designed for vanets. *The Journal of Supercomputing*.

[13] Suárez-Albela M., Fraga-Lamas P., Fernández-Caramés T. (2018). A practical evaluation on RSA and ECC-based cipher suites for IoT high-security energy-efficient fog and mist computing devices. *Sensors*.

[14] Yu M., Zhang J., Wang J. (2018). Internet of Things security and privacy-preserving method through nodes differentiation, concrete cluster centers, multi-signature, and blockchain. *International Journal of Distributed Sensor Networks*.

[15] Braeken A. (2018). PUF based authentication protocol for IoT. *Symmetry*.

[16] Zhou C., Zhao Z., Zhou W., Mei Y. (2017). Certificateless key-insulated generalized signcryption scheme without bilinear pairings. *Security and Communication Networks*.

[17] Kumari S., Karuppiah M., Das A. K., Li X., Wu F., Kumar N. (2017). A secure authentication scheme based on elliptic curve cryptography for IoT and cloud servers. *The Journal of Supercomputing*.

[18] Omala A. A., Mbandu A. S., Mutiria K. D., Jin C., Li F. (2018). Provably secure heterogeneous access control scheme for wireless body area network. *Journal of Medical Systems*.

[19] Tamizhselvan C., Vijayalakshmi V. (2019). An energy efficient secure distributed naming service for IoT. *International Journal of Advanced Studies of Scientific Research*.

[20] Naresh V. S., Sivaranjani R., V.E.S. Murthy N. (2018). Provable secure lightweight hyper elliptic curve-based communication system for wireless sensor networks. *International Journal of Communication Systems*.

[21] Rahman A. U., Ullah I., Naeem M. (2018). A lightweight multi-message and multi-receiver heterogeneous hybrid signcryption scheme based on hyper elliptic curve. *International Journal of Advanced Computer Science and Applications*.

[22] Ta V. D., Liu C.-M., Nkabinde G. W. Big data stream computing in healthcare real-time analytics.

[23] Even S., Goldreich O., Micali S. (1990). On-line/off-line digital signatures. *Advances in Cryptology—CRYPTO’ 89 Proceedings*.

[24] Shamir A., Tauman Y. (2001). Improved online/offline signature schemes. *Advances in Cryptology-CRYPTO 2001*.

[25] Yu P., Tate S. R. Online/offline signature schemes for devices with limited computing capabilities.

[26] Wu T., Chen Y., Lin K. ID-based online/offline signature from pairings.

[27] Addobea A. A., Hou J., Li Q. (2020). MHCOOS: An Offline-Online Certificateless Signature Scheme for M-Health Devices. *Security and Communication Networks*.

[28] Islam S. K. H., Biswas G. P. (2013). Provably secure and pairing-free certificateless digital signature scheme using elliptic curve cryptography. *International Journal of Computer Mathematics*.

[29] Khan M. A., Qureshi I. M., Khanzada F. (2019). A hybrid communication scheme for efficient and low-cost deployment of future flying ad-hoc network (FANET). *Drones*.

[30] Shamus Sofware Ltd. http://github.com/miracl/MIRACL

[31] Khan M. A., Ullah I., Nisar S. (2020). An efficient and provably secure certificateless key-encapsulated signcryption scheme for flying ad-hoc network. *IEEE Access*.

[32] Khan M. A., M Qureshi I., Ullah I., Khan S., Khanzada F., Noor F. (2020). An efficient and provably secure certificateless blind signature scheme for flying ad-hoc network based on multi-access edge computing. *Electronics*.

[33] Khan M. A., Ullah I., Nisar S. (2020). Multiaccess edge computing empowered flying ad hoc networks with secure deployment using identity-based generalized signcryption. *Mobile Information Systems*.

[34] Ullah I., Alomari A., Ul Amin N., Khan M. A., Khattak H. (2019). An energy efficient and formally secured certificate-based signcryption for wireless body area networks with the internet of things. *Electronics*.

